This article has been retracted.

# Analysis of Efflux Pump System and Other Drug Resistance Related Gene Mutations in Tigecycline-Resistant *Acinetobacter baumannii*

**DOI:** 10.1155/2023/8611542

**Published:** 2023-02-17

**Authors:** Wenzheng Zheng, Yubo Huang, Wenbin Wu, Jiaxin Zhu, Tiantuo Zhang

**Affiliations:** Department of Pulmonary and Critical Care Medicine, the Third Affiliated Hospital of Sun Yat-Sen University, Sun Yat-Sen University, and Institute of Respiratory Diseases, Guangzhou 510000, China

## Abstract

**Background:**

The isolation of tigecycline-resistant *Acinetobacter baumannii* in recent years has brought great difficulties to clinical prevention and treatment.

**Purpose:**

To explore the effect of efflux pump system and other resistance related gene mutations on tigecycline resistance in *Acinetobacter baumannii*.

**Methods:**

Fluorescence quantitative PCR was used to detect the expression levels of major efflux pump genes (*adeB*, *adeJ*, and *adeG*) in extensive drug-resistant *Acinetobacter baumannii*. The minimum inhibitory concentration (MIC) of tigecycline was detected by the broth microdilution testing and efflux pump inhibition experiment to assess the role of efflux pump in tigecycline resistance of *Acinetobacter baumannii*. Efflux pump regulatory genes (*adeR* and *adeS*) and tigecycline resistance related genes (*rpsJ*, *trm*, and *plsC*) were amplified by PCR and sequenced. By sequence alignment, tigecycline sensitive and tigecycline-insensitive *Acinetobacter baumannii* were compared with standard strains to analyze the presence of mutations in these genes.

**Results:**

The relative expression of *adeB* in the tigecycline-insensitive *Acinetobacter baumannii* was significantly higher than that in the tigecycline sensitive *Acinetobacter baumannii* (114.70 (89.53-157.43) vs 86.12 (27.23-129.34), *P* = 0.025). When efflux pump inhibitor carbonyl cyanide 3-chlorophenylhydrazone (CCCP) was added, the percentage of tigecycline-insensitive *Acinetobacter baumannii* with tigecycline MIC decreased was significantly higher than that of tigecycline-sensitive *Acinetobacter baumannii* (10/13 (76.9%) vs 26/59 (44.1%)), *P* = 0.032); the relative expression of *adeB* in the MIC decreased group was significantly higher than that in the MIC unchanged group (110.29 (63.62-147.15) vs 50.06 (26.10-122.59), *P* = 0.02); The relative expression levels of efflux pumps *adeG* and *adeJ* did not increase significantly, and there was no significant difference between these groups. One *adeR* point mutation (Gly232Ala) and eight *adeS* point mutations (Ala97Thr, Leu105Phe, Leu172Pro, Arg195Gln, Gln203Leu, Tyr303Phe, Lys315Asn, Gly319Ser) were newly detected. Consistent mutations in *trm* and *plsC* genes were detected in both tigecycline-insensitive and tigecycline-sensitive *Acinetobacter baumannii*, but no mutation in *rpsJ* gene was detected in them.

**Conclusion:**

Tigecycline-insensitive *Acinetobacter baumannii* efflux pump *adeABC* overexpression was an important mechanism for tigecycline resistance, and the mutations of efflux pump regulator genes (*adeR* and *adeS*) are responsible for *adeABC* overexpression. The effect of *trm*, *plsC*, and *rpsJ* gene mutations on the development of tigecycline resistance in *Acinetobacter baumannii* remains controversial.

## 1. Introduction

*Acinetobacter baumannii* (AB) is a nonmotile, oxidase-negative, nonfermenting sugar Gram-negative bacillus [1]. It is highly environmentally adaptable and can survive up to 5 months on dry solid surfaces due to biological properties such as low nutrient requirements, ability to survive in most temperature and pH environments, high resistance to disinfectants, and ease of biofilm formation on nonliving surfaces [2]. At the same time, its intrinsic resistance and its ability to rapidly upregulate endogenous resistance mechanisms or actively acquire exogenous resistance genes allow it to evolve relatively quickly into a multiresistant bacterium with resistance to multiple antibiotics [3]. As a result, *Acinetobacter baumannii* is widely present in health care settings and difficult to eradicate. Extensive drug-resistant *Acinetobacter baumannii* (XDR AB) refers to insusceptibility to all classes of antimicrobial drugs except colistin and tigecycline [4, 5], and several studies have shown that drug-resistant *Acinetobacter baumannii* infections have been shown to have a high mortality rate, especially for carbapenem-resistant *Acinetobacter baumannii* (CRAB) infections, which can range from 35% to 61% [6–11]. Tigecycline (TGC) is currently regarded as an effective drug against CRAB or XDR-AB [12, 13], however, with the gradual application of tigecycline in clinical practice, tigecycline resistant *Acinetobacter baumannii* also emerged in recent years [14–16].

The mechanism of tigecycline resistance production by *Acinetobacter baumannii* is a hot topic of current interest, and existing studies suggest that overexpression of the efflux pump system plays a major role in multidrug resistant bacteria [17–19]. Closely related to *Acinetobacter baumannii* tigecycline is the RND family, which contains three major systems: *adeABC*, *adeFGH*, and *adeIJK* [20]. However, the degree of correlation between overexpression of each system and tigecycline resistance levels may vary, and whether the efflux pump system can play an important role in altering tigecycline resistance levels in clinical strains in which multiple resistance mechanisms may coexist, which issues are still controversial [21–23]. Meanwhile, it has been reported that the variation of *adeRS* two-component system changed the sensitivity of *Acinetobacter baumannii* to tigecycline by regulating the expression of efflux pump system [24, 25]. Moreover, recent studies have identified mutations in tigecycline drug target genes or membrane permeability-related genes in some strains without efflux pump overexpression, such as *trm*, *plsC*, and *rpsJ* genes [26–28], and the prevalence of these resistance genes in clinical drug-resistant strains has been less studied so far. Therefore, we explored the role of the above mechanisms in tigecycline-resistant *Acinetobacter baumannii* in our hospital.

## 2. Materials and Methods

### 2.1. Sources of Strains and Reagents

Seventy-two strains of extensive drug-resistant *Acinetobacter baumannii* isolated from the sputum of patients in the Third Affiliated Hospital of Sun Yat-Sen University from April 2014 to September 2017 were collected for tigecycline resistance mechanism study. The reagents used in our study were as follows: M-H broth dry powder (MUELLER-HINTON BROTH); OXOID, UK, carbonyl cyanide 3-chlorophenylhydrazone (CCCP); Sigma-Aldrich, USA, tigecycline dry powder (standard); Dalian Meilun Biological, China, magnesium chloride anhydrous; Shanghai Maclean, China, calcium chloride anhydrous; Shanghai Maclean, China, diethyl pyrocarbonate (DEPC); Sigma-Aldrich, USA, RNAiso Plus; TaKaRa, Dalian, China, LightCycler 480 SYBR Green I Master; Roche, Switzerland, Transcriptor cDNA Synth. Kit 1: Roche, Switzerland, Isopropanol; Guangzhou Chemical Reagent Factory, China, Chloroform; Guangzhou Chemical Reagent Factory, China, Anhydrous Ethanol; Guangzhou Chemical Reagent Factory, China, Dimethyl Sulfoxide (DMSO); Guangzhou Chemical Reagent Factory, China; Lysozyme; Sigma-Aldrich, USA; M-H Agarase; Sigma-Aldrich, USA. Aldrich; M-H agar dry powder (MUELLER-HINTON AGAR); OXOID, UK; 250 bp DNA Ladder (Dye Plus); and Baobao Bioengineering (Dalian) Co.

### 2.2. Drug Susceptibility Test (Broth Microdilution Method) and Efflux Pump Inhibition Test

The drug susceptibility test adopts the broth microdilution method, referring to the M07-A9 aerobic bacteria dilution method antibacterial drug susceptibility test standard (ninth edition) issued by the CLSI in the United States in 2012 [29]. The efflux pump inhibition test is the drug sensitivity test of TGC combined with CCCP efflux pump inhibitor (10ug/ml). The breakpoint of tigecycline sensitivity is based on the FDA standard: MIC≤2ug/ml is sensitive and MIC≥8ug/ml is resistant. *Escherichia coli* ATCC25922 were used as the drug-susceptible quality control bacteria, and *Acinetobacter baumannii* standard strain ATCC17978 was used as the control bacteria.

### 2.3. RNA Extraction and cDNA Synthesis

Extraction of bacterial total RNA was referred to the recommended steps of TaKaRa's RNAiso Plus (No. 9108/9109) and cDNA synthesis (reverse transcription) was performed according to the steps recommended by Transcriptor cDNA Synth. Kit 1 (No. 04 897 030 001).

### 2.4. Real-Time PCR

The standard strain of *Acinetobacter baumannii* ATCC17978 was used the control strain, and the mRNA expression of the *rpoB* reference gene of each target strain and the three efflux pump systems *adeB*, *adeG*, and *adeJ* of the RND family were detected, and the relative expression of these three efflux pump genes was calculated. Specific steps were as follows:

Synthesis of primer sequences: The primer sequences of target genes *adeB*, *adeG*, *adeJ*, and *rpoB* internal reference genes are shown in Table 1, and the synthesis was commissioned by BGI (Beijing Liuhe) Co.Ltd.

Reaction system and conditions: Follow the steps recommended by LightCycler 480 SYBR Green I Master.

Result data processing: Both the amplification curve and the dissolution curve were single-peak curves, indicating that the product amplification repeatability and specificity were good, and the qualified test data was collected for calculation. mRNA relative expression (RE) = 2^−△△^Ct, where ^△△^Ct = (Ct Target-Ct *rpoB*) target strain-(Ct Target - Ct *rpoB*) control strain.

### 2.5. Detection of Efflux Pump Regulator Gene *adeRS* and Drug Resistance Related Genes *plsC*, *Trm* and *rpsJ*

Preparation of bacterial genomic DNA template is as follows: scrape a ring of fresh monoclonal bacteria cultured on LB agar medium overnight, resuspend in sterilized water, place in a 100°C water bath for 10 min, and collect the supernatant by centrifugation as the strain genomic DNA template.

Synthesis of primer sequences is as follows: the primer sequences of regulatory genes *adeR*, *adeS*, and drug resistance-related genes *plsC*, *trm*, and *rpsJ* are shown in Table 2, and the synthesis was commissioned by BGI (Beijing Liuhe) Co.Ltd.

The target gene amplification was performed in the Applied Biosystems PCR system (Veriti Thermal Cycler) with Golden DNA polymerase (Golden Easy PCR System KT221, TIANGEN BIOTECH (BEIJING), China).

The amplification conditions of the regulated genes *adeR* and *adeS* are shown as follows. The amplification conditions included 35 cycles of amplification under the following conditions: initial denaturation at 94°C for 5 min, denaturation at 94°C for 30 s, annealed at 54°C for 30 s, extend at 72°C for 2 min, and a final extension at 72°C for 5 min.

The amplification conditions of drug resistance-related genes *plsC*, *trm*, and *rpsJ* were shown as follows. Amplification was carried out with the following thermal cycling conditions: 5 min at 94°C and 35 cycles of amplification consisting of 30 s at 94°C, 30 s at 58/56/54°C (for *plsC*/*trm*/*rpsJ*, respectively), and 1 min at 72°C, with 5 min at 72°C for the final extension.

### 2.6. PCR Product Electrophoresis and Gel Imaging

Recovery, purification, and sequencing of PCR products by electrophoresis and gel cutting, BGI (Beijing Liuhe) Co., Ltd. was entrusted to carry out electrophoresis, gel cutting, recovery, and purification of PCR products, and the Sanger method was used for two-way detection and splicing.

Gene sequence alignment submitted the spliced gene sequence fragments to the PubMed website for BLAST alignment and annotated the unknown sequence fragments. Using the *adeR*, *adeS*, *plsC*, *trm*, and *rpsJ* genes in the complete genome of *Acinetobacter baumannii* standard strain ATCC17978 (NZ_CP018664.1) as the reference sequence, Bioedit and SnapGene software were used to perform multiple sequence alignment, translation, and mutation type of each spliced sequence identification.

### 2.7. Statistical Methods

The database was established using SPSS version 21.0 software package and statistical processing was performed. Normally distributed measurement data were described as mean ± standard deviation ($\bar{\text{x}}\pm \text{SD}$), and comparisons were made using independent samples *t*-test; nonnormally distributed measurement data were described as median (25% quantile~75% quantile); and described and compared using rank sum test. *P* < 0.05 difference was statistically significant. Graphs were drawn using GraphPad Prism 7.

## 3. Results

### 3.1. Drug Susceptibility Test and Efflux Pump Inhibition Test

The distribution of tigecycline MIC of 72 extensive drug-resistant *Acinetobacter baumannii* strains was shown in Figure 1, and the range of MIC was distributed between 16-0.5 ug/ml. According to the FDA tigecycline susceptibility criteria (MIC≥8 ug/ml as resistant, MIC≤2 ug/ml as sensitive), these *Acinetobacter baumannii* were divided into two groups: tigecycline sensitive extensive drug-resistant *Acinetobacter baumannii* (TS-XDR AB) group, which tigecycline MIC was less than or equal to 2 ug/ml, and tigecycline insensitive extensive drug-resistant *Acinetobacter baumannii* (TIS-XDR AB) group, which tigecycline MIC was greater than 2ug/ml. Among them, there were 59 strains (81.9%) in TS-XDR AB group and 13 strains (18.1%) in TIS-XDR AB group. The number of MIC 2 and 1 strains was relatively high, with 24 (33.3%) and 28 (38.9%) strains, respectively. This part of the results showed that this TIS-XDR AB accounted for only a small proportion of XDR AB, but they could indeed be isolated from clinical patients, and even individual TIS-XDR AB developed high levels of resistance to tigecycline.

When the efflux pump inhibitor CCCP was added, the statistics of the MIC decreased of tigecycline in *Acinetobacter baumannii* were shown in Table 3 and Figure 2. Among them, the tigecycline MIC of 36 strains decreased by 2-8 times, accounting for 50%, 26 strains (44.1%) were TS-XDR AB, and 10 strains (76.9%) were TIS-XDR AB. The proportion of TIS-XDR AB with tigecycline MIC decreased was higher than that in TS-XDR AB group, which was statistically significant (*P* = 0.032). That is, the tigecycline MIC decreased of the TIS-XDR AB group was inhibited by the efflux pump was significantly higher than the TS-XDR AB group. The tigecycline MIC decreased by more than 2 times, which significantly affected by CCCP, including 6 strains, accounting for about 8.3%, of which 4 strains were TIS-XDR AB, and 2 strains were TIS-XDR AB. This part of the results showed that efflux pump inhibitors play a more important role in reducing tigecycline sensitivity in TIS-XDR AB than in TS-XDR AB.

### 3.2. Analysis of the Relative Expression of Efflux Pump System Detected by Real-Time Quantitative PCR

The relative expression (RE) of three main efflux pump genes was different between the TS-XDR AB group and the TIS-XDR AB group. Statistical analysis, the results are shown in Figure 3.

There is a significant difference in the relative expression of *adeB* gene between these two groups (*P* = 0.025). The relative expression of *adeB* in the TIS-XDR AB group is significantly higher than that in the TS-XDR AB group. However, there was no significant difference in the relative expression of *adeG* and *adeJ* genes between these two groups. This part of the results showed that *adeB* was significantly overexpressed in TIS-XDR AB compared with TS-XDR AB.

### 3.3. Analysis of the Relationship between the Relative Expression of the Efflux Pump System and the Decrease in Tigecycline Sensitivity

Grouping according to the efflux pump inhibition experiment, the RE of three major efflux pump genes was statistically analyzed between the tigecycline MIC decreased group and the tigecycline MIC no changed group, and the results were shown in Figure 4.

It can be seen that there was a significant difference in the RE of *adeB* gene between these two groups; that is, the RE of *adeB* in the tigecycline MIC decreased group is significantly higher than that in the tigecycline MIC no changed group. However, there was no significant difference in the RE of *adeG* and *adeJ* genes between these two groups. This part of the results showed that the overexpression of *adeB* was closely related to the reduction of tigecycline resistance in XDR AB by efflux pump inhibitors.

### 3.4. Amplification and Sequence Alignment of Efflux Pump Regulator Genes *adeR* and *adeS* and Drug Resistance-Related Genes *plsC*, *Trm* and *rpsJ*

The efflux pump regulation genes (*adeR* and *adeS*) and tigecycline resistance related genes (*plsC*, *trm*, and *rpsJ*) of 13 tigecycline insensitive extensive drug-resistant *Acinetobacter baumannii* were detected, and 4 tigecycline sensitive extensive drug-resistant *Acinetobacter baumannii* were used as controls. The tigecycline MIC of these *Acinetobacter baumannii* were shown in Tables 4.

The expected amplified fragments of *adeR* and *adeS* genes are about 800 bp and 1200 bp, and most strains can amplify the corresponding specific target fragments. The electropherogram of some strains were shown in Figure 5. Among them, the target fragments of the *adeS* gene amplified by the four strains 587, 576, 579, and 594 were significantly larger than expected, and the bands were about 2500 bp in Figure 5(b), suggesting that these genes may have inserted sequences.

The expected amplified fragments of *plsC*, *trm*, and *rpsJ* genes are about 1400 bp, 1200 bp, and 300 bp, and each strain can amplify the corresponding specific purpose fragment, the electropherogram of PCR products of some strains were shown in Figure 6.

These 17 extensive drug-resistant *Acinetobacter baumannii* have detected mutations in *adeR* and *adeS* genes, including substitution, insertion mutation, and deletion mutations. The nonsynonymous mutations of each strain were shown in Table 5. It can be seen in the table that there were 5-6 missense mutations in the *adeS* gene of each strain, but only 2-3 missense mutations in *adeR*. Among them, the *adeR* of 511S, 576, and 594 strains had single-base insertions at different sites (Insert652A, Insert718G, Insert32C) resulting in nonsense mutation which is the early appearance of termination codons (229 Stop, 246 Stop, 13 Stop). The translationally synthesized peptide chain was shortened. In addition, the insertion sequence ISAba1 appeared at the 3′ end of the *adeS* of strains 576, 579, 587, and 594, which would affect the transcription of downstream genes. This part of the results showed that several nonsynonymous mutations were detected in *adeR* and *adeS* genes.

These 17 extensive drug-resistant *Acinetobacter baumannii* were found to contain mutations in *plsC*, *trm* genes, including substitution, insertion mutation, and deletion mutation. The nonsynonymous mutations of each strain were shown in Table 5. No mutation was found in the *rpsJ*. There was a missense mutation (CAA592AAA) and a terminator codon mutation (TAA925AAA) in the *plsC* gene. There were insertions or deletions bases at different sites (Insert29A, Deletion51A, Deletion267A) in the *trm* gene, resulting in nonsense mutation which is the early appearance of termination codons (16 Stop, 37 Stop, 92 Stop), and the peptide chain synthesized by translation of the gene was shortened. This part of the results showed that nonsynonymous mutations were detected in both *plsC* and *trm* but not in *rpsJ*.

## 4. Discussion

The efflux pump mechanism is an important mechanism for the resistance of *Acinetobacter baumannii* tigecycline. The RND family is the first reported and widely recognized efflux pump family, including *AdeABC*, *AdeFGH*, and *AdeIJK*. Among them, overexpression of *adeABC* efflux pump system plays the largest role in drug resistance [30–32]. Efflux pump inhibitors restore sensitivity to the drug by inhibiting the active efflux of the *Acinetobacter baumannii* efflux pump.

In this study, the relative expression levels of the multidrug transporter genes *adeB*, *adeG*, and *adeJ* in the efflux pump systems *adeABC*, *adeFGH*, and *adeIJK* of 72 XDR-Aba strains were detected, and it was found that the relative expression levels of *adeB* were significantly increased. Moreover, the relative expression of TIS group was significantly higher than that of TS-XDR group, suggesting that overexpression of *adeB* was closely related to tigecycline resistance in *Acinetobacter baumannii*, and overexpression of *adeB* was the main factor reducing the sensitivity of tigecycline in *Acinetobacter baumannii*. While the relative expression of *adeG* and *adeJ* did not increase significantly, and there was no significant difference between the two groups, suggesting that the expression of these two efflux pump systems is not closely related to the tigecycline resistance of *Acinetobacter baumannii*, and their overexpression is not a cause of reduced tigecycline susceptibility in *Acinetobacter baumannii*. These results are consistent with other reports [21, 33, 34].

The efflux pump inhibition test also confirmed the above inference that after the addition of CCCP, the relative expression of *adeB* in the tigecycline MIC decreased group is significantly higher than that in the tigecycline MIC no changed group, suggesting that overexpression of *adeB* is closely related to the decreased tigecycline sensitivity induced by the inhibition of efflux pump, and overexpression of *adeB* is the main factor that efflux pump inhibitors reduce the tigecycline sensitivity of clinical *Acinetobacter baumannii*. While the relative expression of *adeG* and *adeJ* did not increase significantly, and there was no significant difference between the two groups, suggesting that the expression of these two efflux pump systems is not closely related to the decrease of tigecycline sensitivity due to the inhibition of efflux pumps, and their overexpression is not the reason that efflux pump inhibitors reduce tigecycline sensitivity in *Acinetobacter baumannii*. 50% (36 strains) of the strains showed a 2-8 fold decrease in MIC, suggesting that the active efflux of the efflux pump can increase the tigecycline MIC of most strains. However, only 8.3% (6 strains) of the strains had a greater than 2-fold decrease in MIC, of which 4 were non-susceptible strains, and the proportion of non-susceptible strains was 30.8% (4/13 strains), suggesting that the role of the efflux pump in affecting tigecycline MIC is limited. It is possible that multiple resistance mechanisms may combine to influence the sensitivity of tigecycline. In conclusion, although the efflux pump mechanism may play a limited role, the efflux pump system adeABC was widely present in *Acinetobacter baumannii* [35, 36], which is a fundamental factor for increasing the level of tigecycline resistance, and is even more critical in the resistance mechanism of a small number of strains.

Overexpression of the *adeABC* efflux pump system is regulated by the two-component regulatory gene *adeRS*, and mutations in either the *adeR* or *adeS* genes may lead to *adeABC* expression [37–39]. *adeB* expression was significantly increased in all 13 tigecycline-insensitive strains, and detection of *adeR* and *adeS* genes in these strains revealed by comparison that they had 2-7 nonsynonymous mutations. The *adeS* gene was more prone to mutations than the *adeR* gene, a phenomenon in agreement with the studies of Montana S et al. [40] and Hammerstrom Troy G et al. [41], suggesting that *adeS* has a higher degree of genetic variation and plays a more active role in the regulation of *adeABC* overexpression. Four nonsynonymous point mutations (Val120Ile, Ala136Val, Gly232Ala, Asp20Asn) and one insertional mutation (Insert32C) were found in *adeR* gene, and 12 nonsynonymous point mutations (Ala94Val, Ala97Thr, Leu105Phe, Leu172Pro, Gly186Val Arg195Gln, Gln203Leu, Asn268His, Tyr303Phe, Lys315Asn, Gly319Ser, Val348Ile) and one insertional mutation (ISAba1 inserted at the end of *adeS*) were found in *adeS* gene. In addition to three *adeR* point mutations (Val120Ile, Ala136Val, Asp20Asn) and four *adeS* point mutations (Ala94Val, Gly186Val, Asn268His, Val348Ile) and the insertion of ISAba1 mutation in *adeS* were reported to be associated with *adeABC* overexpression in previous studies [21, 36, 42, 43]; the remaining one *adeR* point mutation (Gly232Ala) and eight *adeS* point mutations (Ala97Thr, Leu105Phe, Leu172Pro, Arg195Gln, Gln203Leu, Tyr303Phe, Lys315Asn, Gly319Ser) were newly detected in this study, and these mutations may lead to elevated expression of *adeABC*, but their specific effects remain to be experimentally verified. In addition to the efflux pump mechanism, some studies in recent years have also reported that mutations in the *trm*, *rpsJ* and *plsC* genes lead to increased tigecycline resistance [26–28]. Therefore, this study detected the sequences of these genes in 13 tigecycline-insensitive strains and 4 tigecycline-sensitive strains, to understand the resistance mechanism of tigecycline-insensitive *Acinetobacter baumannii* in our hospital. *Trm* gene detection found that 17 strains all had single base deletions or insertions (Insert29A, Deletion51A, Deletion267A) at different sites, resulting in nonsense mutation which is the early appearance of stop codons (16 Stop, 37 Stop, 92 Stop) and shortened synthesis. However, 4 of them were tigecycline-sensitive strains with MICs ranging from 0.25 to 1 ug/ml, so it was speculated that *trm* deletion could not significantly improve the resistance of *Acinetobacter baumannii* to tigecycline. This result is different from previous reports that the study compared the whole gene sequence of the tigecycline-insensitive mutant strain and its parental strain by genome sequencing, and found that the *trm* deletion mutation was the only difference between the two. It is speculated that the *trm* gene deletion leads to the decrease of tigecycline sensitivity. Chen Q et al. [27] also found a 35 bp nucleotide deletion in the *trm* gene of the drug-resistant mutant strain by genome sequencing. The wild-type *trm* gene complementation experiment restored the mutant strain's sensitivity to tigecycline, confirming that the *trm* gene mutation is one of the mechanisms of tigecycline resistance in *Acinetobacter baumannii*. Based on the above findings, we believe that *trm* gene deletion leads to tigecycline resistance is still controversial, and more studies are needed to clarify. *plsC* gene detection found that non-synonymous point mutations (Gln198Lys) and terminator codon mutations (Stop309Lys) were also present in tigecycline-sensitive *Acinetobacter baumannii*, suggesting that these mutations could not lead to tigecycline resistance. Although the study by Li X et al. [28] confirmed that the frameshift mutation of the *plsC* gene caused the synthetic shortened peptide chain leading to tigecycline resistance, this study did not detect the *plsC* gene deletion mutation. Therefore, the *plsC* gene deletion mutation is not the cause of the tigecycline resistance in *Acinetobacter baumannii* in our hospital. The *rpsJ* gene detection found that 13 strains did not find any mutation points, indicating that the gene is not related to tigecycline resistance in these strains.

In summary, our study revealed that the expression of *adeABC* efflux pump in extensive drug-resistant *Acinetobacter baumannii* was significantly increased, and the increase was more significant in tigecycline insensitive strains. The overexpression of *adeABC* was closely related to tigecycline resistance, and the mechanism of efflux pump was the cause of tigecycline resistance. It is a common and important mechanism, but only this mechanism has a limited impact, and most strains may have multiple resistance mechanisms that eventually lead to an increase of tigecycline resistance. *AdeABC* overexpression is the result of *adeRS* gene mutation, 1 *adeR* and 8 *adeS* point mutations have not been reported in previous studies, and the relationship between these mutant genes and *adeABC* overexpression remains to be explored. *trm*, *plsC*, and *rpsJ* genes have nothing to do with the resistance of *Acinetobacter baumannii* tigecycline in our hospital. The effect of *trm*, *plsC*, and *rpsJ* gene mutations on the development of tigecycline resistance in *Acinetobacter baumannii* remains unclear. Besides the pump mechanism, there might be other resistance mechanisms.

## Figures and Tables

**Figure 1:** Distribution of tigecycline (TGC) MIC of 72 extensive drug-resistant *Acinetobacter baumannii* strains.

**Figure 2:** Distribution of fold change in tigecycline MIC of *Acinetobacter baumannii* altered by CCCP (carbonyl cyanide 3-chlorophenylhydrazone).

**Figure 3:** Relative expressions (RE) of efflux pump genes (*adeB*, *adeG*, and *adeJ*) of *Acinetobacter baumannii*. TIS-XDR AB: tigecycline insensitive extensive drug-resistant *Acinetobacter baumannii*; TS-XDR AB: tigecycline sensitive extensive drug-resistant *Acinetobacter baumannii*.

**Figure 4:** Relative expressions (RE) of efflux pump genes (*adeB*, *adeG*, and *adeJ*) of *Acinetobacter baumannii*. MIC decreased: the tigecycline MIC decreased group; MIC NC: the tigecycline MIC no changed group.

**Figure 5:** Electropherogram of efflux pump regulation genes *adeR* and *adeS* of *Acinetobacter baumannii* ((a) *adeR* gene, 1-9 were 583, 587, 588, 594, 576, 579, 590S, 591, ATCC17978; (b) *adeS* gene, 1-9 were 583, 587, 588, 594, 576, 579, 590S, 591, respectively, of which 587, 594, 576, 579 target fragments were about 2500 bp, larger than expected fragments, suggesting that there may be an insertion sequence.).

**Figure 6:** Electropherogram of tigecycline resistance-related genes *plsC*, *trm*, and *rpsJ* in *Acinetobacter baumannii* ((a) *plsC* gene, 1-5 were511R, 528, 579, 591, ATCC17978; (b) *trm* gene, 1-4 were498, 502, 507, 512, respectively; (c) *rpsJ* gene, 1-10 were 498, 502, 507, 512, 517, 536, 583, 587, 588, 594, respectively).

**Table 1:** Sequence list of fluorescent quantitative PCR primers.

Gene name	Primer name	Primer sequence(5′-3′)
*rpoB*	*rpoB*-F	TCCGCACGTAAAGTAGGAAC
	*rpoB*-R	ATGCCGCCTGAAAAAGTAAC

*adeB*	*adeB*-F	CTTGCATTTACGTGTGGTGT
	*adeB*-R	GCTTTTCTACTGCACCCAAA

*adeG*	*adeG*-F	GTGTAGTGCCACTGGTTACT
	*adeG*-R	ATGTGGGCTAGCTAACGGC

*adeJ*	*adeJ*-F	GGTCATTAATATCTTTGGC
	*adeJ*-R	GGTACGAATACCGCTGTCA

**Table 2:** List of primer sequences for each target gene.

Gene name	Primer name	Primer sequence(5′-3′)
*adeR*	*adeR*-F	GTTAAGGCAATAAAAAGTTGCTT
	*adeR*-R	TGGAGTAAGTGTGGAGAAATACG

*adeS*	*adeS*-F	CTTGGTTAGGTTAGATATGGCATT
	*adeS*-R	GGCGTGGGATATAGGCTAGATAA

*plsC*	*plsC*-F	CTAGGATCCTACCAGCCATTTGTTCGC
	*plsC*-R	TTGGTCGACCACGGTGATATTTCGTTTGC

*trm*	*Trm*-F	AAGGATCCACTTTATATGAGTCACC
	*Trm*-R	ATAACTGGATCCATCCACTCACCTT

*rpsJ*	*rpsJ*-F	ACCCAAAGCGATCTGAACATCAACAC
	*rpsJ*-R	ATGTCTAACCAGAGAATTCGTATCCGTCTTAAGTC

**Table 3:** TGC MIC decreased of *Acinetobacter baumannii* altered by CCCP.

	XDR AB	TS-XDR AB	TIS-XDR AB	*P*
Total number	72	59	13	
Number of TGC MIC decreased	36	26	10(76.9%)	
Rate of TGC MIC decreased	50%	44.1%	76.9%	0.032^∗^

**Table 4:** TGC MIC of 17 extensive drug-resistant *Acinetobacter baumannii.*

Strain number	498	502	507	511R	517	528	579	583	587	588	591	594
TGC MIC (*μ*g/ml)	4	4	4	16	8	8	8	8	4	4	4	4

Strain number	511S	524	576	590S								
TGC MIC (*μ*g/ml)	0.5	1	1	0.25								

**Table 5:** Base changes of non-synonymous mutations in *adeRS*, *plsC*, *trm*, and *rpsJ* genes of each strain and their corresponding amino acid changes.

Strain number	*adeR*	*adeS*	*plsC*	*Trm*	*rpsJ*
498	GTC358ATC(Val120Ile); GCA407GTA(Ala136Val); GGC695GCC(Gly232Ala)	CTT515CCT(Leu172Pro); GGT557GTT(Gly186Val); AAT802CAT(Asn268His); TAT908TTT(Tyr303Phe); GTT1042ATT(Val348Ile)	CAA592AAA(Gln198Lys); TAA925AAA(Stop309Lys)	Deletion51A(CAA51CAG; Gln17Gln) 37 Stop	None

502	GTC358ATC(Val120Ile); GCA407GTA(Ala136Val); GGC695GCC(Gly232Ala)	CTT515CCT(Leu172Pro); GGT557GTT(Gly186Val); AAT802CAT(Asn268His); TAT908TTT(Tyr303Phe); GTT1042ATT(Val348Ile)	CAA592AAA(Gln198Lys); TAA925AAA(Stop309Lys)	Deletion51A(CAA51CAG; Gln17Gln) 37 Stop	None

507	GTC358ATC(Val120Ile); GCA407GTA(Ala136Val); GGC695GCC(Gly232Ala)	CTT515CCT(Leu172Pro); GGT557GTT(Gly186Val); AAT802CAT(Asn268His); TAT908TTT(Tyr303Phe); GTT1042ATT(Val348Ile)	CAA592AAA(Gln198Lys); TAA925AAA(Stop309Lys)	Deletion267A(ATA267ATG; Ile89Met) 92 Stop	None

511S	GAT58AAT(Asp20Asn); GTC358ATC(Val120Ile); GCA407GTA(Ala136Val); Insert652A(CTG652ACT; Leu218Thr) 229 Stop	CTC313TTC(Leu105Phe); CTT515CCT(Leu172Pro); GGT557GTT(Gly186Val); AAT802CAT(Asn268His); TAT908TTT(Tyr303Phe); GTT1042ATT(Val348Ile)	CAA592AAA(Gln198Lys); TAA925AAA(Stop309Lys)	ATT88CAT(Asn30His); Deletion267A(ATA267ATG; Ile89Met) 92 Stop	None

511R	GAT58AAT(Asp20Asn); GTC358ATC(Val120Ile); GCA407GTA(Ala136Val)	CTC313TTC(Leu105Phe); CTT515CCT(Leu172Pro); GGT557GTT(Gly186Val); AAT802CAT(Asn268His); TAT908TTT(Tyr303Phe); GTT1042ATT(Val348Ile)	CAA592AAA(Gln198Lys); TAA925AAA(Stop309Lys)	Deletion51A(CAA51CAG; Gln17Gln) 37 Stop	None

512	GTC358ATC(Val120Ile); GCA407GTA(Ala136Val)	CTT515CCT(Leu172Pro); GGT557GTT(Gly186Val); CAG608CTG(Gln203Leu); AAT802CAT(Asn268His); TAT908TTT(Tyr303Phe); GTT1042ATT(Val348Ile)	CAA592AAA(Gln198Lys); TAA925AAA(Stop309Lys)	Deletion267A(ATA267ATG; Ile89Met) 92 Stop	None

517	GAT58AAT(Asp20Asn); GTC358ATC(Val120Ile); GCA407GTA(Ala136Val)	CTC313TTC(Leu105Phe); CTT515CCT(Leu172Pro); GGT557GTT(Gly186Val); AAT802CAT(Asn268His); TAT908TTT(Tyr303Phe); GTT1042ATT(Val348Ile)	CAA592AAA(Gln198Lys); TAA925AAA(Stop309Lys)	Insert29A(GTG29GAT; Val10Asp) 16 Stop	None

524	GTC358ATC(Val120Ile); GCA407GTA(Ala136Val)	CTT515CCT(Leu172Pro); GGT557GTT(Gly186Val); AAT802CAT(Asn268His); TAT908TTT(Tyr303Phe); GTT1042ATT(Val348Ile)	CAA592AAA(Gln198Lys); TAA925AAA(Stop309Lys)	Deletion267A(ATA267ATG; Ile89Met) 92 Stop	None

528	GTC358ATC(Val120Ile); GCA407GTA(Ala136Val)	GCC281GTC(Ala94Val); CTT515CCT(Leu172Pro); GGT557GTT(Gly186Val); AAT802CAT(Asn268His); TAT908TTT(Tyr303Phe); GTT1042ATT(Val348Ile)	CAA592AAA(Gln198Lys); TAA925AAA(Stop309Lys)	Deletion51A(CAA51CAG; Gln17Gln) 37 Stop	None

576	GTC358ATC(Val120Ile); GCA407GTA(Ala136Val); Insert718G(CCC718GCC; Pro240Ala) 246 Stop	CTT515CCT(Leu172Pro); GGT557GTT(Gly186Val); AAT802CAT(Asn268His); TAT908TTT(Tyr303Phe); GTT1042ATT(Val348Ile); ISAba1	ACT55CCT(Thr19Pro); CAA592AAA(Gln198Lys); TAA925AAA(Stop309Lys)	Deletion267A(ATA267ATG; Ile89Met) 92 Stop	None

579	GTC358ATC(Val120Ile); GCA407GTA(Ala136Val)	CTT515CCT(Leu172Pro); GGT557GTT(Gly186Val); AAT802CAT(Asn268His); TAT908TTT(Tyr303Phe); AAA945AAT(Lys315Asn); GTT1042ATT(Val348Ile); ISAba1	CAA592AAA(Gln198Lys); TAA925AAA(Stop309Lys)	Deletion267A(ATA267ATG; Ile89Met) 92 Stop	None

583	GTC358ATC(Val120Ile); GCA407GTA(Ala136Val)	GCA289ACA(Ala97Thr); CTT515CCT(Leu172Pro); GGT557GTT(Gly186Val); AAT802CAT(Asn268His); TAT908TTT(Tyr303Phe); GTT1042ATT(Val348Ile)	CAA592AAA(Gln198Lys); TAA925AAA(Stop309Lys)	Deletion267A(ATA267ATG; Ile89Met) 92 Stop	None

587	GTC358ATC(Val120Ile); GCA407GTA(Ala136Val)	CTT515CCT(Leu172Pro); GGT557GTT(Gly186Val); CGG584CAG(Arg195Gln); AAT802CAT(Asn268His); TAT908TTT(Tyr303Phe); GTT1042ATT(Val348Ile); ISAba1	CAA592AAA(Gln198Lys); TAA925AAA(Stop309Lys)	Deletion267A(ATA267ATG; Ile89Met) 92 Stop	None

588	GTC358ATC(Val120Ile); GCA407GTA(Ala136Val)	GCA289ACA(Ala97Thr); CTT515CCT(Leu172Pro); GGT557GTT(Gly186Val); AAT802CAT(Asn268His); TAT908TTT(Tyr303Phe); GTT1042ATT(Val348Ile)	CAA592AAA(Gln198Lys); TAA925AAA(Stop309Lys)	Deletion51A(CAA51CAG; Gln17Gln) 37 Stop	None

590S	GTC358ATC(Val120Ile); GCA407GTA(Ala136Val)	CTT515CCT(Leu172Pro); GGT557GTT(Gly186Val); AAT802CAT(Asn268His); TAT908TTT(Tyr303Phe); GGC955AGC(Gly319Ser); GTT1042ATT(Val348Ile); ACC1048GCC(Thr350Ala)	CAA592AAA(Gln198Lys); TAA925AAA(Stop309Lys)	Deletion267A(ATA267ATG; Ile89Met) 92 Stop	None

591	GTC358ATC(Val120Ile); GCA407GTA(Ala136Val)	CTT515CCT(Leu172Pro); GGT557GTT(Gly186Val); AAT802CAT(Asn268His); TAT908TTT(Tyr303Phe); GGC955AGC(Gly319Ser); GTT1042ATT(Val348Ile)	CAA592AAA(Gln198Lys); TAA925AAA(Stop309Lys)	GAG135GAC(Glu45Asp); Deletion267A(ATA267ATG; Ile89Met) 92 Stop	None

594	Insert32C(CAA32CCA; Gln11Pro) 13 Stop	CTT515CCT(Leu172Pro); GGT557GTT(Gly186Val); CGG584CAG(Arg195Gln); AAT802CAT(Asn268His); TAT908TTT(Tyr303Phe); GTT1042ATT(Val348Ile); ISAba1	CAA592AAA(Gln198Lys); TAA925AAA(Stop309Lys)	Deletion267A(ATA267ATG; Ile89Met) 92 Stop	None

## Data Availability

The datasets during the current study are available from the corresponding author on reasonable request.
